# Overexpression of SCAMP3 is an indicator of poor prognosis in hepatocellular carcinoma

**DOI:** 10.18632/oncotarget.22665

**Published:** 2017-11-27

**Authors:** Xinyuan Zhang, Jie Sheng, Yuhong Zhang, Yu Tian, Jie Zhu, Nan Luo, Congshu Xiao, Rongkuan Li

**Affiliations:** ^1^ Department of Infection, The Second Hospital of Dalian Medical University, Dalian, Liaoning, P.R. China; ^2^ Department of Nephrology, The Second Hospital of Dalian Medical University, Dalian, Liaoning, P.R. China; ^3^ Department of Ultrasound, The Second Hospital of Dalian Medical University, Dalian, Liaoning, P.R. China; ^4^ Division of Hepatobiliary and Pancreatic Surgery, Department of Surgery, The Second Hospital of Dalian Medical University, Dalian, Liaoning, P.R. China; ^5^ Clinical Laboratory of the Second Hospital of Dalian Medical University, Dalian, Liaoning, P.R. China

**Keywords:** hepatocellular carcinoma, secretory carrier membrane protein 3, prognosis

## Abstract

SCAMP3, an isoform of the secretory carrier membrane proteins (SCAMPs) family, is a membrane-trafficking protein involved in endosome transport. Previous microarray data showed that SCAMP3 mRNA is highly expressed in hepatocellular carcinoma (HCC). In this study, the expression and clinical significance of SCAMP3 in 100 pairs of HCC and adjacent normal tissue were investigated. siRNA transfection was performed to silence SCAMP3 expression in HCC cells. The MTS assay and flow cytometry were used to detect the proliferation, cell cycle progression of HCC cells. Compared with adjacent normal tissues, SCAMP3 expression was dramatically increased in HCC tissues demonstrated by Western blotting (*P* < 0.05). In immunohistochemistry, compared with the adjacent normal tissues, SCAMP3 was detected in 96% of the HCC samples with a significant increase in intensity and number of stained cells (*P* < 0.05). Also, high SCAMP3 expression was found in 86% of the HCC samples (*P* < 0.05). The increased SCAMP3 expression was significantly correlated with vascular invasion (*P* = 0.004) and tumor stage (*P* = 0.001). Univariate and multivariate survival analyses showed that the expression of SCAMP3 was an independent prognostic factor of overall survival of HCC patients. Knockdown of SCAMP3 expression led to suppression of cell proliferation and blockage of cell cycle of HCC cells. In conclusion, our present study suggested that SCAMP3 may serve as a promising prognostic biomarker and molecular target of HCC and further investigation is warranted.

## INTRODUCTION

The liver cancer is the most common primary malignancy of the liver and it is the sixth most common cancer worldwide [1]. Hepatocellular carcinoma (HCC) accounts for more than 80% of primary liver cancers. While more than 80% of HCC occurred in sub-Saharan Africa and Eastern Asia, and the incidence has risen in the Western countries [2]. And almost half of the new cases and related deaths of HCC occurred in China [3]. Although great progress has been achieved in treatment techniques for HCC, the prognosis of HCC patients is still poor. Due to high rates of recurrence and metastasis, long-term survival after radical surgical resection is still unsatisfactory [4, 5]. Hepatocarcinogenesis has a complicated course, which presents with a series of genetic and epigenetic changes that occur during initiation, promotion, and progression of the disease. These changes include gene mutations, modifications of oncogenes and tumor-suppressor genes, copy number variations and gene rearrangements, epigenetic modifications and alterations in numerous signaling pathways [6-8]. Although considerable efforts and large molecular studies have been undertaken to elucidate the mechanism of hepatocarcinogenesis, the latter still remains unclear. Secretory carrier membrane proteins (SCAMPs) are a family of integral membrane proteins ubiquitously expressed across taxa and which are predominantly located in secretory membranes [9-11]. Although the function of SCAMPs is not yet known, several previous studies suggested that SCAMPs may play a crucial role in exocytosis and vesicle budding in mammalian cells [12-14]. These studies showed that SCAMPs, like pantophysin, jointly existed in recycling transport vesicles comprising of post-Golgi and endocytic pathways, and the SCAMPs may mainly take effect at the same location during vesicular transport rather than in separate post-Golgi recycling pathways [14]. But studies on relationships between SCAMPs and tumors, which were reported in SCAMP1and SCAMP3 were rare [15-17]. The previous study, in which cDNA microarrays were used to characterize patterns of gene expression in HCC, demonstrated that SCAMP3 was highly expressed in HCC tissue compared to those seen in non-tumor liver tissues [18]. Another study has shown that chromosome band 1q22 was the commonly involved region in HCC with eight genes detected in both significance analysis of microarray and gene set enrichment analysis [19]. SCAMP3 was one of those eight genes located in 1q22 and was significantly up regulated in both mathematical models [19]. Those previous studies emphasized the importance of SCAMP3 and supported a hypothesis that SCAMP3 may play a role in the pathogenesis of HCC. In this study, we investigated the role of SCAMP3 in human HCC cells. We used Western blotting and immunohistochemistry to investigate the expression of SCAMP3 both in HCC and the adjacent normal liver tissue. We also analyzed the relationship between SCAMP3 expression and clinicopathological features. The prognostic value of SCAMP3 was determined in HCC patients. In addition, the effect of SCAMP3 knockdown in cell cycle and cell proliferation of HCC cells were investigated.

## RESULTS

### SCAMP3 is up regulated in HCC tissues

Western blotting analysis was performed to investigate the SCAMP3 expression between 100 pairs of matched HCC tissues and the adjacent normal ones. The result showed that the expression of SCAMP3 was dramatically increased in HCC tissues compared with the adjacent normal tissues (Figure 1A). And the expression of SCAMP3 protein was dramatically up regulated in 94% (94/100) of HCC samples. The ratio of SCAMP3 expression to GAPDH was displayed in a bar chart showing a significant higher expression of SCAMP3 in HCC tissues than in the adjacent normal tissues (Figure 1B, ^*^P < 0.01).

**Figure 1:** The expression of SCAMP3 in HCC and adjacent normal tissues **(A)** The protein levels of SCAMP3 in HCC (T) and adjacent normal tissues (N) were determined by western blotting in 100 paired samples. SCAMP3 expression was significantly increased in HCC (T) compared with the adjacent normal tissues (N). Representative images of eight paired samples were shown. GAPDH was used as a control. **(B)** The bar chart shows the ratio of SCAMP3 protein to GAPDH by densitometry, showing a significant higher expression of SCAMP3 in HCC tissues than in the adjacent normal tissues. The data are mean ± SEM of three independent experiments (^*^P < 0.01, HCC tissues to adjacent normal tissues).

The expression of SCAMP3 in 100 pairs of HCC tissues and adjacent normal tissues were evaluated by immunohistochemical analysis. SCAMP3 was mainly expressed in the cytoplasm (Figure 2). The expression of SCAMP3 was higher in HCC specimens than adjacent normal ones (Figure 2A-2D). The rate of the SCAMP3 positive cells were calculated by immunohistochemical evaluation as previously described. The expression of SCAMP3 in HCC was found in 96% (96/100) of samples, which was significantly higher than that of the adjacent normal tissues (8%, 8/100) (*P* < 0.05). According to the previous principle of IHC staining score, the expression of SCAMP3 was divided into two grades: high SCAMP3 expression and low SCAMP3 expression. High SCAMP3 expression was found in 86% of the HCC samples, which was significantly higher than that of the adjacent normal tissues (2%, 2/100) (*P* < 0.05).

**Figure 2:** Immunohistochemical analysis of SCAMP3 expression in HCC and adjacent normal tissues Paraffin-embedded HCC tissue sections were stained with antibodies against SCAMP3 and counterstained with hematoxylin. **(A, B)** Low expression of SCAMP3 in the adjacent normal tissues (SP, A, ×100; B, ×400). **(C, D)** High SCAMP3 expression in HCC Specimen (SP, C, ×100; D, ×400).

### The correlation between SCAMP3 expression and clinicopathological parameters in HCC

The correlation of SCAMP3 expression and clinicopathologic parameters was analyzed. The clinicopathological parameters of patients were summarized in Table 1. The results showed that SCAMP3 expression was significantly correlated with vascular invasion (*P* = 0.004) and tumor stage (*P* = 0.001). No significant correlation was found between SCAMP3 expression and other clinicopathological features including age, gender, hepatitis B antigen, liver cirrhosis, tumor size, tumor differentiation and AFP (Table 1).

**Table 1:** Correlation of clinicopathological parameters and SCAMP3 expression

Variable	SCAMP3			
	All cases	Low expression	High expression	*P* value
**Age, y**				1.000
<55	47	7	40	
≥55	53	7	46	
**Gender**				1.000
Male	84	12	72	
Female	16	2	14	
**Hepatitis B ag**				0.726
Positive	81	11	70	
Negtive	19	3	16	
**Cirrhosis**				1.000
Yes	78	11	67	
No	22	3	19	
**Tumor size, cm**				1.000
≥5	36	5	31	
<5	64	9	55	
**Vascular invasion**				**0.003**
Present	**67**	**4**	**63**	
Absent	**33**	**10**	**23**	
**Tumor differentiation**				0.571
Well	7	1	6	
Moderate	61	11	50	
Poor	32	2	30	
**Tumor stage**				**0.028**
I-II	**63**	**13**	**50**	
III-IV	**37**	**1**	**36**	
**AFP, ng/ml**				0.114
<20	30	7	23	
≥20	70	7	63	

### Increased SCAMP3 expression predicts poor prognosis in HCC patients

Kaplane-Meier survival analyses were applied to determine the prognostic value of SCAMP3 in HCC. The results showed that the patients with high expression of SCAMP3 tended to have worse survival (Figure 3A and 3B). Furthermore, the Cox’s proportional hazards Regression model showed that the expression of SCAMP3 (*P* = 0.001), tumor size (*P* = 0.011) and vascular invasion (*P* = 0.000) were independent prognostic factors of overall survival (Table 2).

**Figure 3:** High SCAMP3 expression is associated with poor prognosis of patients with HCC **(A)** Kaplan–Meier survival curves showed the significant differences in overall survival. **(B)** Recurrence-free survival between the HCC patients with high and low SCAMP3 expression (all *P* < 0.05, log-rank test).

**Table 2:** Cox regression analysis

Parameters	Hazard ratio	95% confidence interval	*P* value
tumor size	2.007	1.176-3.424	0.011
vascular invasion	3.945	2.220-7.007	0.000
SCAMP3 expression	3.532	1.670-7.469	0.001

### Knockdown of SCAMP3 affected cell proliferation and cell cycle of HCC cells

In order to study the potential effects of SCAMP3 on HCC cell proliferation, the endogenous SCAMP3 was knocked down in Huh7, PLC5 and Hep3B cells by RNA interference. All the cell lines were transfected with SCAMP3-siRNA. The efficiencies of RNA interference were evaluated by Western blotting assay. The protein level of SCAMP3 was dramatically decreased in transfected with SCAMP3-siRNA cells compared with the control siRNA transfected cells (Figure 4A, Figure 4C and Figure 4E). MTS assay was used to determine the effect of knockdown of SCAMP3 on cell proliferation of Huh-7, PLC5 and Hep3B cells. The average absorbance value of the SCAMP3-siRNA cell groups were significantly lower compared with the NC group after transfection of SCAMP3-siRNA at 48 hr and 72 hr (all *P* < 0.05) (Figure 4B, Figure 4D and Figure 4F). The effects of SCAMP3 knockdown on cell cycling progression was further analyzed by flow cytometry. The results of flow cytometry analysis revealed that Huh-7, PLC5 and Hep3B cells in SCAMP3-siRNA groups were arrested in G1 phase (Figure 5A-5C).

**Figure 4:** Knockdown of SCAMP3 expression affected cell proliferation of HCC cell linesHuh7, PLC5 and Hep3B **(A-F)** Western blotting analyses of knockdown efficiency of SCAMP3-targeting siRNA oligos of Huh7 (A), PLC5 (C) and Hep3B (E) cells and proliferation of Huh7 (B), PLC5 (D) and Hep3B (F) cells was significantly suppressed in SCAMP3-siRNA groups compared with NC groups.

**Figure 5:** Knockdown of SCAMP3 expression affected cell cycle of HCC cell lines **(A-C)** The proportions of Huh7 (A), PLC5 (B), Hep3B (C) cells in G1 phase increased significantly in SCAMP3-siRNA group in comparison with NC group.

## DISCUSSION

In SCAMPs family, there are four distinct isoforms including SCAMP1-4, which are ubiquitously expressed in mammalian cells, and the fifth isoform (SCAMP5) exhibits primarily neural expression. In structure, all SCAMPs have a highly conserved tetraspanning transmembrane core named SCAMP domain, and the domain is centrally located and comprises of four hydrophobic transmembrane domains (TMDs) with three inter-TMD-flanking sequences [11]. The hydrophilic loop between transmembrane span 2 and 3 forms the E-peptide which shows the highest degree of sequence conservation across taxa. The cytoplasmic N- and C-termini, flanking the SCAMP domain, show different length and highest diversity over taxa [11]. These cytosolic peptides harbor distinct protein-protein interacting motifs which are important for SCAMPs function and localization, and the SCAMP domain is indispensable for its correct targeting [20-23]. The transcriptional units (Tus) involving SCAMP3 may represent a genuine novel transcript indispensable in keeping pluripotency of the embryonic stem (ES) cell [24]. Also, SCAMP3 is regarded as an important component of Salmonella-induced filaments (SIFs) and SCAMP3 tubules manipulate specific post-Golgi trafficking which may allow Salmonella to obtain nutrients or to regulate host immune responses [25]. In addition, SCAMP3 plays a role in sorting and budding of intraluminal vesicles and is involved in the process of multivesicular endosome biogenesis [14]. Moreover, SCAMP3 is regarded as a positional and functional candidate gene for type 2 diabetes (T2DM) [26].

In this study, we disclosed the SCAMP3 expression in human HCC tissue and the adjacent normal liver tissue, along with its correlation with the clinicopathological parameters. We demonstrated that SCAMP3 expression was higher in human HCC tissue either by Western blotting or IHC compared to the adjacent normal liver tissue. SCAMP3 expression was significantly correlated with vascular invasion, tumor stage and poor survival. Furthermore, from *in vitro* study, our results showed that knockdown of SCAMP3 by siRNA induced suppression of cell proliferation, caused HCC cells to be arrested at G1 phase. The HCC cell lines included Huh-7, PLC5 and Hep3B cells. Although the mechanism is not clear, our results suggested that SCAMP3 may contribute to the pathogenesis and progression of HCC. To the best of our knowledge, this is the first time to study the SCAMP3 expression both in human HCC tissue and HCC cell lines, with correlation to clinicopathological features and survival data of the HCC patients, has been done. The previous study by Naboulsi Wet al., analyzed 36 tissue specimens from HCC patients by quantitative proteomics and showed that thirty endocytosis-associated proteins were mostly overexpressed in poorly differentiated tumors which included SCAMP3 [17]. Their continuous studies also revealed that the expression of SCAMP3 was immunohistochemically increased in tissue sections of 84 HCC patients. But the study lacked the analysis of the clinicopathological features and survival data with SCAMP3 expression.

The receptor-mediated endocytosis is essential to activate the abundance of membrane receptors through recycling and degradation [27]. And, endocytosis would be helpful in providing fresh signaling receptors to the plasma membrane and important for cancer progression via activating the recycling of tumorigenic receptors or preventing their degradation, which eventually cause a consistent oncogenic activation of the associated tumorigenic pathways [28-30]. The SCAMPs members have rarely been reported in association with malignant tumors at protein level before. Previous studies have demonstrated that the expression of SCAMP1, the isoform of SCAMPs family, was different (up-regulated) between the cervical cancer tissues from the patients with and without lymphatic metastasis, which indicated that SCAMP1 may be involved in the process of lymphatic metastasis of cervical cancer [15]. Moreover, SCAMP1 was also reported to be highly expressed in both human pancreatic and gallbladder cancer cells [16]. And SCAMP1 could be regarded as the potential targeted gene for treatment of pancreatic and gallbladder cancer [17]. It was shown that down regulation of SCAMP1 inhibited vascular endothelial growth factor (VEGF) activity in both human pancreatic and gallbladder cancer cell lines. The high level of VEGF activation was significantly associated with advanced tumor stage and lymphatic metastasis, which subsequently involved the alterations of a series of genes, including some oncogenes and tumor suppressor genes, such as K-ras, c-myc, c-fos, c-erbB-2, p53, p16 and deleted in pancreatic cancer, locus 4 (DPC4). Those abnormal changes played an important role in the development and progression of the pancreatic cancer [31]. However, how endocytic protein SCAMP3 is involved in pathogenesis and progression of HCC is not clear, but speculations can be made. Previous studies showed that SCAMP3 played an important role in regulation of epidermal growth factor receptor (EGFR) degradation [32, 33]. EGFR is a transmembrane receptor tyrosine kinase that can be activated by several ligands and is related to some signaling pathways, controlling mainly proliferation, differentiation and survival [34-36]. Several studies have demonstrated that EGFR overexpression was found in 68% of human HCCs and correlated with aggressive tumors, metastasis, and poor survival [37-40]. The EGFR signaling system was regarded as a key role in the liver response to injury which include early inflammation, hepatocellular proliferation, fibrogenesis and neoplastic transformation, which facilitate the genetic alterations leading to unrestrained cell proliferation and development of HCC [41]. Therefore, we speculate that SCAMP3 may be involved in pathogenesis and progression of HCC via EGFR and its signaling system. Such a speculation has also been addressed by Naboulsi Wetet al. [17]. Aoh et al. [33] demonstrated that knockdown of SCAMP3 accelerated EGFR degradation. However, there is no direct evidence to show EGFR protein level in the presence and absence of SCAMP3 using immunoassays-based analysis. In our knockdown experiments, we found SCAMP3 knockdown did not change the EGFR level in Huh7 and Hep3B HCC cells by western blotting (data not shown). Thus, SCAMP3 function in HCC still remains unknown.

In conclusion, our study showed that the expression of SCAMP3 was up-regulated in human HCC tissue, and the up-regulated SCAMP3 was closely related to vascular invasion, tumor stage and indicated poor survival of HCC. In addition, the knockdown of SCAMP3 decreased cell proliferation and cell cycle progression of HCC cells. These data suggest that SCAMP3 may serve as a promising prognostic biomarker and molecular target of HCC. However, further study to clarify the mechanism of SCAMP3 in the pathogenesis and progression of HCC is warranted.

## MATERIALS AND METHODS

### Patients and specimens

100 surgically treated HCC patients were enrolled in the study and all HCC specimens were collected at the Second Affiliated Hospital of Dalian Medical University at Dalian in China between January 2010 and January 2016. All HCC specimens were collected according to the protocols approved by the local ethical committee. All patients gave their written informed consent to participation in the study. HCC specimens and the adjacent normal tissue were harvested during surgery. None of the patients had received any adjuvant therapies prior to surgery. The clinical and pathologic parameters of the patients were collected for analysis and were shown in Table 1. All samples were immediately processed after surgical resection for further analysis. According to the Edmondson-Steiner grading system, tumor differentiation was graded as follows: well differentiated, moderately differentiated and poorly differentiated. The tumor stage was defined according to the Barcelona Clinic Liver Cancer (BCLC) staging system [42]. Overall survival (OS) was the interval between surgery and the date of death; and recurrence-free survival (RFS) was the interval between surgery and the date of recurrence. All patients were followed till July 2016 and the follow-up time was between 6–66 months (median, 37.5 months).

### Cell line culture and siRNA transfection

Human liver cancer cell lines Huh-7 was obtained from JCR Bank. PLC5 and Hep3B were obtained from ATCC. The cell lines were maintained in Dulbecco’s modified eagle’s medium (DMEM, Gibco, USA) supplemented with 10% fetal bovine serum (FBS, Gibco, USA) and 100 units/mL penicillin and 100 μg/mL streptomycin, in the presence of 5% CO_2_ at 37 °C. A SCAMP3-specific predesigned siRNA (ID 19579, Targeting sequence: GCU ACU CGA CAG AAC AA UUT T) and silencer negative control siRNA were purchased from Thermo Fisher Scientific. All procedures of the transfection assays were performed with RNAiMAX reagent (Invitrogen, MA, CA) according to the manufacturer’s instructions. Western blotting assay was used to evaluate the efficiency of the knockdown.

### Western blotting

Total protein was extracted from tissues or harvested cells using T-PER Tissue Protein Extraction Reagent with protease inhibitor cocktail and phosphatase inhibitor cocktail (Pierce; Rockford, IL), and protein concentration was determined with BCA Protein Assay Kit (Pierce, Rockford, IL). Equal amounts of protein (20μg) were electrophoresed on 4% to 12% polyacrylamide gels (Invitrogen, Carlsbad, CA), and transferred onto PVDF membranes, blocked with 10% nonfat milk for at least 1 hour, and probed with primary antibodies against SCAMP3 (1:1000, Cat #:PA5-21428, Thermo Fisher Scientific, CA) and GAPDH (1:1000, SC-365062, Santa Cruz, CA).

The specific proteins were detected with HRP-conjugated secondary antibodies (Santa Cruz Biotechnology; Santa Cruz, CA) and SuperSignal West Pico or West Femto Maximum Sensitivity substrate from Pierce (Rockford, IL). The ratio of SCAMP3/GAPDH was used to assess the protein expression level.

### Immunohistochemistry (IHC) and evaluation

Two-step immunohistochemical method was used and performed for the immunostaining according to the manufacturer’s instructions. HCC tissue sections were embedded in paraffin and were dewaxed in xylene and graded alcohols, hydrated, and washed in PBS. Antigen retrieval was performed by 0.01mol/L of citrate buffer (pH 6.0) and a microwave. Endogenous peroxidase activity was blocked by 3% hydrogen peroxide (in fresh methanol) for 10 min at room temperature. After washing with phosphate-buffered saline (PBS), the sections were incubated with a blocking serum for 1h. Then, the slides were stained with primary polyclonal rabbit antibodies against SCAMP3 (1:500, Cat #:PA5-21428, Thermo Fisher Scientific, CA) for the whole night at 4°C. After washing in PBS, the sections were incubated with a secondary antibody, horseradish peroxidase (HRP)-labeled goat anti-rabbit IgG (Thermo Fisher Scientific, CA). Positive staining was displayed with DAB. SCAMP3 protein expression was examined independently by two experienced investigators. The percentage of positive tumor cells was counted in five separate fields with 1000 cells randomly selected and scored. The percentage of positively stained cells was scored as “0” (<10%), “1” (10–30%), “2” (30–50%), “3” (50–70%) and “4” (>70%). The intensity of staining was scored as follows: “0” (negative staining); “1” (weak staining); “2” (moderate staining); and “3” (strong staining). The immunostaining score was calculated by multiplying the percentage score by the staining intensity score, ranging from 0 to 12. For statistical analysis, the samples were grouped as negative (score ≤3) and positive (score > 3). And 0–4 was regarded as low expression, while 5–12 were regarded as high expression.

### Cell cycle analysis

The cells were harvested and were fixed in 70% ethanol overnight at 4°C. The fixed cells were treated with 0.25% Triton X-100 for 5 min in an ice bath and stained in a propidium iodide solution (50μg/ml, sigma, USA) which contained 0.1 mg/ml RNase. The cell suspension was incubated in the dark for 30 min at room temperature. Then cell cycle analysis was performed by FACScan flow cytometer (BD Biosciences, Bedford, MA). And the percentages of cells in G1, S, and G2/M phases of the cell cycle were determined from three independent experiments.

### MTS assay

The cell viability was determined by MTS assay. The cells transfected with control siRNA and SCAMP3 siRNA were seeded at a density of 6×10^3^ cells/well in a 96-well culture plates (100 μl/well). After the treatment, CellTiter96® AqueousOne Solution Cell Proliferation Assay (Promega, Madison, Wisconsin) were used according to the manufacturer’s instructions. The absorbance values at 490 nm were detected to determine the number of viable cells and five parallels were set for each well. The absorbance values were analyzed for 24 h, 48 h and 72 h after transfection.

### Statistical analysis

Statistical analyses were performed using the SPSS 19.0 software (SPSS, Chicago, IL, USA). Wilcoxon matched paired test was used to determine the significance of SCAMP3 in HCC and the adjacent normal tissues. A *χ*^2^ test was performed to analyze the correlation between SCAMP3 expression and clinicopathological parameters. Kaplan-Meier curves and the log-rank test were used in analyzing the survival data. Cox proportional hazards regression model was used to identify the independent prognostic factors. A value of *P*<0.05 was considered statistically significant.
